The article "Quercetin Inhibits Tumorigenesis of Colorectal Cancer Through Downregulation of hsa_circ_0006990" was retracted in 2023. Reasons: results that could not be reproduced; contaminated cell lines or tissues.

# Quercetin Inhibits Tumorigenesis of Colorectal Cancer Through Downregulation of hsa_circ_0006990

**DOI:** 10.3389/fphar.2022.874696

**Published:** 2022-05-18

**Authors:** Bin Chen, Linguangjin Wu, Xiaoxia Tang, Ting Wang, Shuyun Wang, Hongjie Yu, Guangsheng Wan, Manli Xie, Ruijuan Zhang, Haijuan Xiao, Wanli Deng

**Affiliations:** ^1^ Department of Oncology, Putuo Hospital, Shanghai University of Traditional Chinese Medicine, Shanghai, China; ^2^ Department of Traditional Chinese Medicine, Putuo People’s Hospital, Tongji University, Shanghai, China; ^3^ Department of Oncology, Affiliated Hospital of Shaanxi University of Chinese Medicine, Xianyang, China

**Keywords:** tumor-associated macrophages, quercetin, hsa_circ_0006990-miR-132-3p/miR-342-3p network, autophagy, colorectal cancer

## Abstract

Quercetin can significantly inhibit the progression of colorectal cancer (CRC). However, its specific mechanism remains largely unclear. In this study, we aimed to explore the correlation among quercetin, tumour-associated macrophages (TAMs) and circular RNAs (circRNAs) in the progression of CRC and to present a novel strategy for the treatment of CRC. In this study, we revealed that quercetin could suppress the autophagy of M2-TAMs and induced their differentiation into M1-TAMs, by which quercetin significantly reversed the inhibition of M2-TAMS on CRC cell apoptosis and the promotion of M2-TAMS on CRC cell proliferation. Moreover, quercetin could promote the expression of downregulated hsa_circ_0006990 in CRC cells co-cultured with M2-TAMs, and the overexpression of hsa_circ_0006990 significantly reversed the anti-tumour effect of quercetin on CRC. Furthermore, we found quercetin can notably suppress the progression of CRC via mediation of the hsa_circ_0006990/miR-132-3p/MUC13 axis. In conclusion, our results suggested that quercetin inhibits the tumorigenesis of CRC *via* inhibiting the polarisation of M2 macrophages and downregulating hsa_circ_0006990. Our study provides useful insights for those exploring new methods of treating CRC.

## Introduction

Colorectal cancer (CRC) is the third most common malignancy in the world (Sung et al., 2021). Moreover, genetic mutations, inflammation-pertinent malfunctions and bad habits may all lead to the progression of CRC (Ferlay et al., 2015; Vasen et al., 2015). Although great efforts have been made in the treatment of CRC, the present situation remains unsatisfactory (Ulaganathan et al., 2018). Therefore, there is an urgent need to explore new strategies for dealing with CRC.

Quercetin is a natural bioflavonoid compound extracted from Hippophae rhamnoides, and it can significantly inhibit the progression of multiple cancers. For example, Mohammed et al. (2021) found that quercetin induced the apoptosis and inhibited the invasion of breast cancer cells; Soofiyani et al. (2021) indicated that quercetin acted as a novel agent for the treatment of lymphoma. Quercetin has also been shown to be able to inhibit the growth of CRC cells (Qi et al., 2021). However, the specific mechanism by which quercetin regulates the progression of CRC remains largely unclear.

Tumour-associated macrophages (TAMs) account for up to 30–50% of total cells in tumour tissues (Coussens and Werb., 2002; Pollard, 2004) and can promote the metastasis and lymphangiogenesis of malignant tumours through recruiting abundant monocytes into the tumour matrix (Pan et al., 2020; Salmaninejad et al., 2019). For instance, TAMs-secreted epidermal growth factor (EGF), PDGF, TGF-β and basic fibroblast growth factor (bFGF) are expected to increase the growth and invasion of tumour cells (Rigo et al., 2010). More importantly, TAMs may exhibit the anti-tumour function by preventing macrophages from converting into type II TAMs (M2-TAMs) (Corthay et al., 2005; Haabeth et al., 2011; Porta et al., 2015). It has also been reported that the inhibition of autophagy inhibits the polarisation of M2-TAMs (Chen et al., 2011) and that the autophagy of TAMs affects the biological activity of CRC cells (Shao et al., 2016). Thus, TAM autophagy may affect the progression of CRC by the regulation of TAM polarisation (Chen et al., 2014). Nevertheless, the exact correlation between quercetin and TAM autophagy in the progression of CRC still needs to be explored experimentally.

Circular RNAs (circRNAs) are endogenous RNAs that have a stable closed structure (Cocquerelle et al., 1993). In addition, it has been reported that circRNAs modulate the cellular processes (cell proliferation, apoptosis, autophagy, etc.) (Jeck et al., 2013; Xia et al., 2017). Meanwhile, circRNAs regulate the growth of CRC cells through sponging miRNAs (Guo et al., 2014; Pervouchine, 2019). For example, hsa_circ_0026344 positively regulates the deterioration of CRC through sponging miR-21/miR-31 (Yuan et al., 2018). However, circRNAs involved in quercetin-mediated CRC progression require further exploration.

Based on the above background, we sought to investigate the correlation among quercetin, TAMs and circRNAs in the progression of CRC and to present a novel strategy for the treatment of CRC.

## Materials and Methods

### Cell Culture

THP-1 cells were obtained from ATCC (United States). Cells were cultured in an incubator at 37 °C and 5% CO_2_. THP-1 cells were maintained in RPMI 1640 medium containing 10% foetal bovine serum (FBS) and 0.05 mmol/L β-mercaptoethanol. CRC cell lines (HCT116 and LoVo) were purchased from the Shanghai Cell Bank of the Chinese Academy of Sciences. They were seeded in RPMI-1640 medium supplemented with 10% FBS. CRC cells were cultured at 37°C and 5% CO_2_.

### Induction and Collection of M2-TAMs

THP-1 cells were seeded into 6-well plates at 1×10^6^/ml density. After treatment with 100 ng/ml PMA for 6 h, THP-1 cells were treated with 20 ng/ml IL-4 for another 18 h. Then, THP-1 cells were cultured with 2 ml fresh serum-free medium for 24 h. The supernatant was subsequently collected to be frozen at -80 °C for later use. The expression of CD68, CD163 and CD206 was identified by flow cytometry.

### Treatment of M2-TAMs With Quercetin

Quercetin (Sigma, United States) was dissolved in dimethyl sulfoxide (DMSO) and then stored at -20 °C for later use. Subsequently, M2-TAMs were treated with quercetin.

### Co-Culture of M2-TAMs and CRC Cell Lines

CRC cells at the logarithmic growth phase were seeded into 6-well culture plates at 1×10^5^/ml density, and M2-TAMs were seeded into the upper transwell chamber (semipermeable membrane pore size: 0.4 μm, model: 3,450, Costar) at 2×10^5^/ml density. Then, CRC cells were treated with the chamber. After 48 h of incubation, total RNAs and proteins were extracted from CRC cells.

### Monodansylcadaverine (MDC) Staining

MDC staining was performed to determine the autophagic vesicles (AVs) of M2-TAMs according to (Biederbick et al., 1995).

### Cell Transfection

CRC cells were seeded into 6-well plates. When the confluence reached 40%, cells were transfected by si-has_circ_0006990/NC, miR-132-3p inhibitor/mimic, miR-342-3p inhibitor/mimic or miR-NC for 48 h using Lipofectamine 2000.

### Colony Formation Assay

CRC cells were seeded into 6-well plates for 12 days. Then, cells were fixed with 4% paraformaldehyde for 15 min and stained with Giemsa solution for 20 min after rinsing with PBS. Finally, the data were calculated.

### TUNEL Assay

Cells were washed and permeabilised. Then, TUNEL reaction mixtures (50 μl) were used to incubate the cells for 60 min with no light. After that, peroxidase (POD, 50 μl) was used to incubate the slides for 30 min at 37°C. Then, cells were rinsed with PBS, and a diaminobenzidine (DAB, 50 μl) substrate solution was used to incubate the cells for 10 min. Finally, the expression of apoptotic cells was observed under an optical microscope.

### Wound Healing Assay

CRC cell lines (1.0×10^5^/ml) were seeded overnight. Then, cells were underlined perpendicular to the cell culture plate with a small pipette head. After washing with PBS three times, serum-free medium was used for further culture, and the scratch widths were recorded at 0 and 24 h under an optical microscope.

### Transwell Invasion Assay

Matrigel (100 μl) was used to pre-treat the upper chamber. CRC cells (1.0×10^6^ cells per chamber) were seeded into the upper chamber in medium (1% FBS). In addition, the lower chamber was supplemented with RPMI1640 (10% FBS). Subsequently, the chamber was rinsed and fixed at 4°C. Then, crystal violet (0.1%) was used to stain the chamber for 20 min. The data were observed under a microscope after the chamber was washed.

### Western Blotting

RIPA was applied to extract proteins from cell lines. A BCA kit was applied to quantify Table 1 the total proteins. SDS-PAGE (10%) was applied to separate the proteins (40 μg per lane), and then proteins were transferred onto PVDF membranes. Subsequently, the membranes were incubated overnight at 4°C with primary antibodies targeted against Bcl-2 (1:1,000), Bax (1:1,000), MUC13 (1:1,000), E2F1 (1:1,000) and GAPDH (1:1,000) after blocking with skimmed milk (5%) for 1 h. Following primary incubation, HRP-conjugated secondary antibodies (1:5,000) were used to incubate the membranes for 1 h. An ECL kit was used to visualise the protein bands. GAPDH was regarded as the internal control. The densitometry analysis was performed using IPP 6.0 (Image-Pro Plus 6.0).

**TABLE 1:** Screening of oncogenic circRNAs in CRC.

CircRNAs	Gene Symbol	Position^a^	Genomic length^a^	Spliced length^a^	Expression Change in CRC	References
hsa_circ_0096088	MACROD1	chr11:63918710–63919865	1,155	219	↑	[PMID: 32564659]
hsa_circ_0006990	VAPA	chr18:9931806–9937063	5,257	338	↑	[PMID: 32564659]
hsa_circ_0004380	TRAPPC9	chr8:141407718–141415797	8,079	248	↑	[PMID: 32564659]
hsa_circ_0001946	CDR1	chrX:139865339–139866824	1,485	1,485	↑	[PMID: 32508871]

a CircBase (http://circrna.org/).

### Real-Time Polymerase Chain Reaction (RT-qPCR)

TRIzol^®^ reagent was applied to extract total RNA. A PrimeScript RT reagent kit was used in reverse transcription. Then, a SYBR Premix Ex Taq II kit (Takara) was used in RT-qPCR, and Real-Time qPCRs were used three times: 2 min at 94 °C, followed by 35 cycles (94 °C for 30 s and 55 °C for 45 s). Primers of circRNAs and miRNAs are listed in Table 2 and Table 3. The data were quantified using the 2^−ΔΔCt^ method. GAPDH was regarded as the internal control.

**TABLE 2:** Primers of colorectal cancer-relevant circRNAs.

CircRNAs	Primers	
	Sense	Anti-sense
hsa_circ_0096088	5′-TGG​AGG​AGC​CCA​GGT​ATA​AA-3′	5′-TCC​ATG​TCG​GGA​TCT​TCT​TC-3′
hsa_circ_0006990	5′-TGA​AAT​GCC​CAA​TGA​AAA​TG-3′	5′-GGC​GAG​GTG​CTG​TAG​TCT​TC-3′
hsa_circ_0004380	5′-GAA​TGC​GGG​AGT​GAT​TGA​GT-3′	5′-TCT​TAG​CAC​GTC​CGA​TCT​CA-3′
hsa_circ_0001946	5′-CAT​GTC​TTC​CAA​CGT​CTC​CA-3′	5′-CTG​GAA​GAC​CCG​GAG​TTG​T-3′

**TABLE 3:** Primers of hsa_circ_0006990-sponged miRNAs.

MiRNAs	Primers	
	Sense	Anti-sense
hsa-miR-3611	5′-GCG​GCG​GTT​GTG​AAG​AAA​GAA​A-3′	5′-ATC​CAG​TGC​AGG​GTC​CGA​GG-3′
hsa-miR-377-3p	5′-GCG​GCG​GAT​CAC​ACA​CAA​AGG​C-3′	5′-ATC​CAG​TGC​AGG​GTC​CGA​GG-3′
hsa-miR-342-3p	5′-GCG​GCG​GTC​TCA​CAC​AGA​AAT​C-3′	5′-ATC​CAG​TGC​AGG​GTC​CGA​GG-3′
hsa-miR-132-3p	5′-GCG​GCG​GTA​ACA​GTC​TAC​AGC​C-3′	5′-ATC​CAG​TGC​AGG​GTC​CGA​GG-3′

### Dual Luciferase Reporter Gene Assay

Hsa_circ_0006990 containing the binding sites of miR-132-3p/miR-342-3p was cloned into the pmirGLO vectors for the establishment of hsa_circ_0006990 (WT/MT). Hsa_circ_0006990 (WT/MT) was transfected into CRC cells with miR-132-3p/miR-342-3p/NC mimics using Lipofectamine 2000. The Dual-Glo Luciferase Assay System was used to analyse the results.

3′-UTR of E2F1/MUC13 containing the putative binding sites of miR-342-3p/miR-132-3p was obtained from Beyotime (Shanghai, China). It was cloned into the pmirGLO vectors to construct wild-type/mutant-type vectors E2F1/MUC13 (WT/MT). E2F1/MUC13 (WT/MT) was transfected into cells using Lipofectamine 2000 (Thermo Fisher Scientific). The Dual-Glo Luciferase Assay System was used to analyse the results.

### Statistical Analyses

Three independent experiments were performed in each group. In addition, the mean ± standard deviation (SD) was used to express all data. The comparisons between two groups were analysed using Student’s t-test, and the differences between multiple groups (more than two) were analysed by one-way analysis of variance (ANOVA) followed by Tukey’s test (Graphpad Prism7). *p* < 0.05 indicates statistical significance.

## Results

### Quercetin Suppressed Polarisation of M2-TAMs *via* Inhibiting Autophagy

THP-1 cells were treated with PMA and IL-4 to induce THP-1 cells into M2-TAMs. As revealed in Figure 1A, cells exhibited more pseudopods and round shapes, which is consistent with the features of M2-TAMs after 48-h treatment (Yunna et al., 2020). Furthermore, the percentages of CD68, CD163 and CD206 in THP-1 cells were significantly increased by PMA and IL-4 (Figure 1B). These data indicate that THP-1 cells were successfully induced into M2-TAMs.

**FIGURE 1:** Quercetin suppressed polarisation of M2-TAMs *via* inhibiting autophagy. **(A)** THP-1 cells were treated with PMA and IL-4. THP-1 cells were observed using a light microscope. **(B)** The percentages of CD68, CD163 and CD206 in THP-1 cells were determined using flow cytometry. **(C)** M2-TAMs were treated with rapamycin, bafilomycin A1 (bafilomycin) or quercetin. The autophagy of M2-TAMs was observed using MDC staining. **(D)** The percentages of CD68 and CD206 in M2-TAMs were measured using flow cytometry.

Additionally, the MDC staining data revealed that the autophagy of M2-TAMs was promoted by rapamycin, while it was obviously inhibited by bafilomycina1 and quercetin (Figure 1C). Meanwhile, bafilomycin A1 and quercetin notably decreased the percentages of CD163 and CD206 (Figure 1D). Taken together, quercetin suppressed the autophagy of M2-TAMs and induced the differentiation into M1-TAMs.

### Quercetin Significantly Reversed M2-TAMs-Induced Proliferation of CRC Cells *via* Inhibiting Autophagy

A colony formation assay was performed after CRC cells were co-cultured with M2-TAMs. The data revealed that the proliferation of CRC cells was significantly promoted by M2-TAMs, which was further increased by rapamycin (Figure 2A). In contrast, M2-TAMs-induced CRC cell proliferation was significantly reversed in the presence of bafilomycin A1 and quercetin (Figure 2A). Moreover, quercetin and bafilomycin A1 greatly induced the apoptosis of M2-TAMs-treated CRC cells (Figure 2B). Meanwhile, M2-TAMs significantly inhibited the level of Bax and upregulated the expression of Bcl-2 in CRC cells, while this phenomenon was greatly restored by bafilomycin A1 and quercetin (Figures 2C,D). In summary, quercetin significantly reversed the M2-TAMs-induced proliferation of CRC cells *via* inhibiting autophagy.

**FIGURE 2:** Quercetin significantly reversed M2-TAMs-induced proliferation of CRC cells *via* inhibiting autophagy. THP-1 cells were treated with PMA and IL-4 and then co-cultured with M2-TAMs (THP-1 cells treated with PMA and IL-4). **(A)** The proliferation of CRC cells was measured using a colony formation assay. **(B)** The apoptosis of CRC cells was tested using TUNEL staining. **(C,D)** The protein levels of Bax and Bcl-2 in CRC cells were investigated using western blotting. GAPDH was used for normalisation. *p < 0.05, **p < 0.01 compared to control. ^#^ *p* < 0.05, ^##^ *p* < 0.01 compared to PMA + IL-4.

### Quercetin Significantly Restored M2-TAMs-Induced Migration and Invasion of CRC Cells *via* Inhibiting Autophagy

To test the effect of M2-TAMs and drug intervention on CRC cell migration, a wound healing assay was used. As shown in Figure 3A, M2-TAMs significantly promoted the migration of CRC cells, while the effect of M2-TAMs was obviously reversed by bafilomycin A1 and quercetin. Consistently, M2-TAMs-induced CRC cell invasion was notably inhibited by bafilomycin A1 and quercetin (Figure 3B). In summary, quercetin significantly restored the M2-TAMs-induced migration and invasion of CRC cells *via* inhibiting their autophagy.

**FIGURE 3:** Quercetin significantly reversed M2-TAMs-induced CRC cell invasion *via* inhibiting autophagy. **(A)** The migration of CRC cells was tested using a wound healing assay. **(B)** The invasion of CRC cells was measured using a transwell assay. *p < 0.05 compared to control. ^#^ *p* < 0.05 compared to PMA + IL-4.

### Quercetin Regulated hsa_circ_0006990 in M2-TAMs-Induced CRC Cells

The differentially expressed circRNAs in CRC are presented in and Supplementary Figure S1A. Among these differentially expressed circRNAs, hsa_circ_0006990 was reported to regulate the tumorigenesis of CRC (Li et al., 2019). Thus, we selected hsa_circ_0006990 for the experiment. Furthermore, downstream miRNAs of hsa_circ_0006990, as predicted by a bioinformatics tool (https://circinteractome.nia.nih.gov/rna_binding_protein.html), were also measured in CRC cells (Supplementary Figure S1B). It was indicated that miR-132-3p and miR-342-3p were both downregulated in CRC cells co-cultured with M2-TAMs. In addition, quercetin and bafilomycin A1 reversed the effect of M2-TAMs on miR-132-3p and miR-342-3p levels (Supplementary Figure S1B). Based on the above results, miR-132-3p and miR-342-3p were selected in our study.

The level of miR-132-3p/miR-342-3p in CRC cells was significantly upregulated by miR-132-3p/miR-342-3p mimics but was inhibited by miR-132-3p/miR-342-3p inhibitor (Supplementary Figures S2A,B). Meanwhile, the luciferase activity in WT-hsa_circ_0006990 was significantly reduced by miR-132-3p/miR-342-3p mimics (Supplementary Figures S2C,D). Furthermore, the expression of miR-132-3p and miR-342-3p in CRC cells was negatively regulated by hsa_circ_0006990 (Supplementary Figures 2E, F).

### Quercetin Inhibited Proliferation and Invasion of CRC Cells *via* Mediation of hsa_circ_0006990

RT-qPCR was performed to investigate the effect of quercetin on hsa_circ_0006990 expression. As demonstrated in Figure 4A, quercetin significantly inhibited the level of hsa_circ_0006990 in CRC cells. In addition, the inhibitory effect of quercetin on CRC cell proliferation was significantly reversed by pcDNA3.1-hsa_circ_0006990 (Figure 4B). Consistently, the overexpression of hsa_circ_0006990 significantly reversed quercetin-induced cell apoptosis (Figure 4C). Furthermore, the migration and invasion of CRC cells was significantly inhibited by quercetin, which was obviously restored by pcDNA3.1-hsa_circ_0006990 (Figures 5A,B). All this shows that quercetin inhibits the proliferation and invasion of CRC cells *via* the mediation of hsa_circ_0006990.

**FIGURE 4:** Quercetin inhibited proliferation of CRC cells *via* mediation of hsa_circ_0006990. **(A)** CRC cells were treated with quercetin. Then, the expression of hsa_circ_0006990 in CRC cells was investigated using RT-qPCR. **(B)** The proliferation of CRC cells was tested using a colony formation assay. **(C)** The apoptosis of CRC cells was tested using TUNEL staining. **p < 0.01 compared to control. ^##^ *p* < 0.01 compared to quercetin.

**FIGURE 5:** Quercetin inhibited migration and invasion of CRC cells *via* mediation of hsa_circ_0006990. **(A)** The migration of CRC cells was tested using a wound healing assay. **(B)** The invasion of CRC cells was tested using a transwell assay. **p < 0.05 compared to control. ^##^ *p* < 0.01 compared to quercetin.

### MiR-342-3p Directly Targeted E2F1 in CRC Cells

To explore the downstream mRNA of miR-342-3p, TargetScan was used. As revealed in Figure 6A, miR-342-3p had binding sites with E2F1, and the luciferase activity in WT-E2F1 was notably decreased by miR-342-3p mimics (Figure 6B). Meanwhile, miR-342-3p negatively regulated the level of E2F1 in CRC cells (Figure 6C). Furthermore, the effect of hsa_circ_0006990 silencing on the E2F1 level was markedly reversed by miR-342-3p inhibitor (Figure 6D). Therefore, MiR-342-3p directly targets E2F1 in CRC cells.

**FIGURE 6:** MiR-342-3p directly targeted E2F1 in CRC cells. **(A)** The downstream target of miR-342-3p was predicted using TargetScan. **(B)** The relative luciferase activity in WT/MUT-E2F1 was tested using a dual luciferase assay. **(C)** CRC cells were transfected with miR-342-3p mimics/inhibitors. Then, the protein level of E2F1 in CRC cells was investigated using western blotting. GAPDH was used for normalisation. **(D)** CRC cells were treated with NC, si-hsa_circ_0006990 or si-hsa_circ_0006990 + miR-342-3p inhibitor. Then, the protein level of E2F1 in CRC cells was investigated using western blotting. GAPDH was used for normalisation. **p < 0.01 compared to control. ^##^ *p* < 0.01 compared to si-hsa_circ_0006990.

### MiR-132-3p Directly Targeted MUC13 in CRC Cells

We also used TargetScan to explore the downstream mRNA of miR-132-3p. As shown in Figure 7A, miR-132-3p had binding sites with MUC13, and the miR-132-3p mimics significantly decreased the luciferase activity in WT-MUC13 (Figure 7B). Meanwhile, miR-132-3p negatively regulated the level of MUC13 in CRC cells (Figure 7C). Furthermore, the effect of hsa_circ_0006990 silencing on MUC13 level was markedly reversed by miR-132-3p inhibitor (Figure 7D). Altogether, MiR-132-3p directly targets MUC13 in CRC cells.

**FIGURE 7:** MiR-132-3p directly targeted MUC13 in CRC cells. **(A)** The downstream target of miR-132-3p was predicted using TargetScan. **(B)** The relative luciferase activity in WT/MUT-MUC13 was tested using a dual luciferase assay. **(C)** CRC cells were transfected with miR-132-3p mimics/inhibitors. Then, the protein level of MUC13 in CRC cells was investigated using western blotting. GAPDH was used for normalisation. **(D)** CRC cells were treated with NC, si-hsa_circ_0006990 or si-hsa_circ_0006990 + miR-132-3p inhibitor. Then, the protein level of MUC13 in CRC cells was investigated using western blotting. GAPDH was used for normalisation. **p < 0.01 compared to control. ^##^ *p* < 0.01 compared to si-hsa_circ_0006990.

## Discussion

Quercetin has been reported to inhibit the progression of malignant tumours (including breast cancer, ovarian cancer and gastric cancer) (Zhou et al., 2016; Liu et al., 2017; Nguyen et al., 2017). The present study found that quercetin also inhibits the progression of CRC. Moreover, this research revealed that quercetin inhibits the M2 polarisation of macrophages as well as their autophagy. Thus, this study firstly explored the function of quercetin in M2-TAMs and autophagy during the progression of CRC, suggesting that quercetin acts as an inhibitor in M2-TAMs.

It has been confirmed that M2-TAMs play a vital role in the tumour microenvironment (Qian and Pollard 2010; Chen and Bonaldo, 2013). For instance, cytokines generated by M2-TAMs (including TNF-α and TGF-ß) induce angiogenesis in breast cancer (Bingle et al., 2006), and the activation of M2-TAMs leads to poor prognosis among patients with tumours (lymphoma, breast cancer, etc.) (Dave et al., 2004; Paik et al., 2004). Consistently, our data showed that quercetin inhibits the tumorigenesis of CRC *via* inhibiting the polarisation of M2 macrophages. On the other hand, it has been reported that autophagy activation leads to the polarisation of macrophages (Yang S. et al., 2021; Yang Y. et al., 2021). The present research indicates that autophagy induces the polarisation of M2 macrophages and that quercetin inhibits the autophagy in M2 macrophages. Thus, it could be suggested that quercetin inhibits the polarisation of M2 macrophages *via* inhibiting their autophagy. Notably, the mechanism by which quercetin regulates the autophagy of M2-TAMs remains unclear, and it needs to be further explored in future.

The present study found that hsa_circ_0006990 was upregulated in CRC cells co-cultured with M2-TAMs. It has been indicated that hsa_circ_0006990 acts as a promoter in CRC [27]. Thus, our data were consistent with this previous study. In addition, our study firstly explored the relation between quercetin and hsa_circ_0006990 in CRC, suggesting that quercetin inhibits the tumorigenesis of CRC *via* the downregulation of hsa_circ_0006990. Meanwhile, the exact correlation among hsa_circ_0006990, M2-TAMs and autophagy requires further investigation.

MiR-342-3p and miR-132-3p were found to be sponged by hsa_circ_0006990 in the present study. In addition, this is the first experiment to elucidate the relation between hsa_circ_0006990 and miR-342-3p/miR-132-3p in CRC. Furthermore, miR⁃342⁃3p/E2F1 and miR-132/MUC13 were also found to be involved in quercetin-mediated CRC progression. It has been reported that miR⁃342⁃3p inhibits the progression of lung cancer (Xue et al., 2018), prostate cancer (Hu et al., 2018), osteosarcoma (Zhang et al., 2017), glioma (Wang et al., 2012) and CRC (Weng et al., 2016; Zhang et al., 2019). Furthermore the downregulation of E2F1 was reported to enhance the sensitivity of CRC cells to oxaliplatin treatment (Fang et al., 2018). Based on those findings, it could be concluded that quercetin significantly inhibits the tumorigenesis of CRC *via* mediation of the hsa_circ_0006990/miR-342-3p/E2F1 axis. On the other hand, miR-132-3p has been reported to act as an inhibitor in cancer progression. That is, miR-132-3p inhibits the progression of lung cancer (Su et al., 2020), glioma (Wang et al., 2018), pituitary tumour (Renjie and Haiqian, 2015), CRC (Zheng et al., 2014) and bladder cancer (Wei and Lv, 2019). More importantly, high-expression miR-132-3p sensitises CRC cells to Adriamycin treatment (Liu and Zhang, 2019). In addition, MUC13 was identified to be the downstream target of miR-132, and it was confirmed to be upregulated in CRC tissues (Walsh et al., 2007). Thereby, our data confirm that quercetin notably suppresses the progression of CRC *via* mediation of the hsa_circ_0006990/miR-132-3p/MUC13 axis.

In conclusion, quercetin inhibits the tumorigenesis of CRC *via* inhibiting the polarisation of M2 macrophages and downregulating hsa_circ_0006990. Thus, the present study provides useful insights for those exploring new methods of treating CRC.

## Data Availability

The raw data supporting the conclusion of this article will be made available by the authors, without undue reservation.

## Supplementary Material

Supplementary Figure S1 Quercetin regulated hsa_circ_0006990 in M2-TAMs-induced CRC cells. **(A)** CRC cells were co-cultured with M2-TAMs. The differentially expressed circRNAs were presented. **(B)** The differentially expressed miRNAs (downstream of has_circ_0006990) were presented.

Supplementary Figure S2 Quercetin regulated hsa_circ_0006990 in M2-TAMs-induced CRC cells. **(A)** CRC cells were transfected with miR-132-3p mimics/inhibitors. The level of miR-132-3p in CRC cells was tested using RT-qPCR. ∗*p*<0.05 compared to miR-NC. **(B)** CRC cells were transfected with miR-342-3p mimics/inhibitors. The level of miR-342-3p in CRC cells was tested using RT-qPCR. **p*<0.05 compared to miR-NC. **(C)** MiR-132-3p was predicted to be the downstream miRNA of hsa_circ_0006990. The relative luciferase activity of WT-hsa_circ_0006990 was measured using a dual luciferase assay. ∗*p*<0.05. **(D)** MiR-132-3p was predicted to be the downstream miRNA of hsa_circ_0006990. The relative luciferase activity of WT-hsa_circ_0006990 was measured using a dual luciferase assay. ∗*p*<0.05. **(E,F)** CRC cells were transfected with si-hsa_circ_0006990 or pcDNA3.1-hsa_circ_0006990. The level of miR-132-3p or miR-342-3p in CRC cells was tested using RT-qPCR. ∗*p*<0.05.

## Glossary

CRC: Colorectal cancer
M2-TAMs: M2 tumour-associated macrophages
TAMs: Tumour-associated macrophages
MDC: Monodansylcadaverine
RT-qPCR: Real-time polymerase chain reaction
EGF: Epidermal growth factor
bFGF: Basic fibroblast growth factor
circRNAs: Circular RNAs
FBS: Foetal bovine serum
DMSO: Dimethyl sulfoxide
AVs: Autophagic vesicles
POD: Peroxidase
DAB: Diaminobenzidine
SD: Standard deviation
ANOVA: Analysis of variance
